The article "NK Cell Subpopulation Is Altered and the Expression of TLR1 and TLR9 Is Decreased in Patients with Acute Lymphoblastic Leukemia" was published in 2021. Journal: J Oncol.

# NK Cell Subpopulation Is Altered and the Expression of TLR1 and TLR9 Is Decreased in Patients with Acute Lymphoblastic Leukemia

**DOI:** 10.1155/2021/5528378

**Published:** 2021-09-15

**Authors:** David Sánchez-Herrera, Alejandra Contreras-Ramos, Elva Jiménez-Hernández, Aurora Medina-Sansón, Silvia Giono-Cerezo, Carmen Maldonado-Bernal

**Affiliations:** ^1^Unidad de Investigación en Inmunología y Proteómica, Hospital Infantil de México Federico Gómez, Secretaría de Salud, Dr. Márquez 162, Col. Doctores 06720, Mexico City, Mexico; ^2^Laboratorio de Biología del Desarrollo, Hospital Infantil de México Federico Gómez, Secretaría de Salud, Dr. Márquez 162, Col. Doctores 06720, Mexico City, Mexico; ^3^Hospital Pediátrico Moctezuma, Gobierno del Distrito Federal, Servicio de Oncología, Secretaría de Salud, Oriente 158, # 189 Col. Moctezuma 2a Sección 15530, Venustiano Carranza, Mexico City, Mexico; ^4^Unidad de Alta Especialidad, Hospital General del Centro Médico Nacional “La Raza”, Instituto Mexicano del Seguro Social, Calzada Vallejo Eje 1 Pte. #208, Azcapotzalco, Mexico City, Mexico; ^5^Unidad de Hemato-Oncología, Hospital Infantil de México Federico Gómez, Secretaría de Salud, Dr. Márquez 162, Col. Doctores 06720, Mexico City, Mexico; ^6^Departamento de Microbiología, Escuela Nacional de Ciencias Biológicas, Instituto Politécnico Nacional, Prolongación de Carpio y Plan de Ayala s/n Col, Casco de Santo Tomás 11340, Mexico City, Mexico

## Abstract

NK cells represent a heterogeneous subpopulation of lymphocytes of the innate immune system, which possess powerful antitumor activity. NK cells exhibit their function through a complex collection of receptors that act synergistically to recognize, regulate, or amplify the immune response. TLRs allow cells to detect PAMPs, MAMPs, or DAMPs, which are essential for the initiation of the immune response. Studies on the different subpopulations of NK cells and their expression profile of innate immune receptors in hematological cancers are limited. In this study, the specific subpopulations of NK cells in pediatric patients with acute lymphoblastic leukemia (ALL) and the repertoire and level of expression of TLRs in cytotoxic NK cells were assessed. The results suggested that pediatric patients with ALL exhibited a significant decrease in NK cells in peripheral blood and bone marrow, in addition to alterations in the distribution of the subpopulations of cells. Regulatory and cytotoxic NK cells were diminished, whereas dysfunctional phenotype was considerably increased. Cytotoxic NK cells from children with ALL expressed all 10 TLRs, and expression of TLR1 and TLR9 was decreased compared with the controls. Interestingly, cytotoxic NK cells exhibited a higher expression of TLR1 in the bone marrow than in the peripheral blood of patients with ALL. The present study is the first to show that TLR10 was expressed in the cytotoxic NK cells and the first to assess the profile and levels of the 10 known TLRs in cytotoxic NK cells from patients with ALL. The alterations in expression levels and cellular distribution may be involved in the immune response.

The article "NK Cell Subpopulation Is Altered and the Expression of TLR1 and TLR9 Is Decreased in Patients with Acute Lymphoblastic Leukemia" was published in 2021. Journal: J Oncol.

## 1. Introduction

Natural killer (NK) cells represent a subpopulation of lymphocytes that participate in the early defense against foreign pathogens or compromised host cells subjected to stress (bacterial infection, viral infection, or tumoral transformation) through their cytotoxic activity or through the production of cytokines and chemokines that generate a proinflammatory environment [1, 2]. NK cells represent 5–15% [3] or even 20% [4] of the mononuclear cells present in the peripheral blood and are phenotypically defined by the expression of CD56 (NCAM) and CD16a (Fc*γ*-RIIIA), but not CD3 and CD19 [5]. Given the expression of CD56, NK cells can be divided into NK^dim^ (cytotoxic) and NK^bright^ (regulatory) subtypes, and, according to coexpression with CD16 and its distribution in peripheral blood or lymphoid organs, it is possible to stratify NK cells into 5 subpopulations with different functional characteristics [6].

The function of NK cells is determined by their phenotype and by a complex collection of receptors that act synergistically to recognize, regulate, or amplify the response to a given stimulus, highlighting the role of pattern recognition receptors (PRRs), such as Toll-like receptors (TLRs) or natural cytotoxicity receptors (NCR), and killer immunoglobulin-like receptors (KIR), such as receptors which direct the early response against pathogens, virally transformed cells, or tumor cells [7].

NK cells play an important role in the innate and adaptive immune responses since their stimulation promotes direct cytotoxic activity on the target cells and/or the rapid release of cytokines and chemokines that initiate the inflammatory process and amplify the adaptive immune response [8].

Despite the fact that the role of NK cells in oncological processes (elimination, editing, and evasion) has been widely discussed both in solid tumors [9] and in hematological cancers [10], relatively little is known about the diversity of the subpopulations of these cells in cancers such as childhood ALL.

Acute lymphoblastic leukemia (ALL) is the most common pediatric malignancy in childhood constituting slightly less than one-third of all childhood cancers diagnosed, while in adolescents and young adults, it constitutes approximately 10% of cancers diagnosed [11].

The article "NK Cell Subpopulation Is Altered and the Expression of TLR1 and TLR9 Is Decreased in Patients with Acute Lymphoblastic Leukemia" was published in 2021. Journal: J Oncol.

Peripheral blood NK cells from patients with acute lymphoblastic leukemia (ALL) type B exhibit compromised cytotoxicity towards K562 and autologous blasts mediated by TGF-*β*1. Furthermore, NKs were found to have an inhibitory phenotype, represented by altered cell surface expression of NKp46 and NKG2A, compared with those from healthy control subjects of the same age [12].

On the other hand, Toll-like receptors (TLRs) are among the most important group of pattern recognition receptors (PRRs), since they orchestrate a wide variety of activities related to the immune response. These receptors recognize a wide variety of molecules evolutionarily conserved, associated with microorganisms, known as pathogen-associated molecular patterns (PAMPs) [13]. TLRs also recognize endogenous molecules called damage-associated molecular patterns (DAMPs), which originate from damaged cells [14] or are products of altered metabolism of transformed cells in conditions such as cancer [15, 16].

Initially, the identification TLR expression in NK cells was based on mRNA detection only. In NK cells isolated from human peripheral blood, the constitutive expression of TLR1-8 mRNA was observed, of which TLRs 2 and 3 were the most abundantly expressed. The expression of TLR9 and 10 mRNA was insignificant in CD56^bright^ and CD56^dim^ NK cell populations [17]. Furthermore, TLR2 mRNA was reported to be highly expressed in resting human NK cells, while TLRs 4 and 3 mRNA were weakly expressed, and TLR8 was undetectable [18]. Additionally, the mRNA levels of these four TLRs increased considerably after exposure to viral particles [18]. Generally speaking, it has been observed that TLRs 2, 3, 5, and 6 are more frequently expressed than TLRs 4, 7, 8, and 9 [19].

Little is known about the expression profile of innate immune response receptors in leukemia, such as TLRs, whose study in NK cells has produced contrasting and controversial results, even in healthy individuals. To the best of our knowledge, there are no studies that have shown whether there is a change in the expression of NK cell TLRs in patients with ALL; the majority of the available studies have focused on studying the changes that exist in infectious diseases, primarily of viral and bacterial diseases [8, 20, 21].

Therefore, in the present study, the frequency of different subpopulations of NK cells as well as the profile and expression levels of TLRs in NK CD16+ cells was determined.

## 2. Materials and Methods

### 2.1. Patients

Nineteen pediatric patients recently diagnosed with ALL, who had not received any prior treatment or transfusions of blood components and were not complicated with infections, were recruited. Peripheral blood samples were taken from nine patients and bone marrow aspirates from the remaining ten.

The article "NK Cell Subpopulation Is Altered and the Expression of TLR1 and TLR9 Is Decreased in Patients with Acute Lymphoblastic Leukemia" was published in 2021. Journal: J Oncol.

The study also included ten peripheral blood samples from healthy individuals who visited the hospital for orthopedic or ophthalmological reasons and who were not complicated by infections and were not immunodeficient.

The present study was approved by the Research, Ethics, and Biosafety Committees of the Children Hospital of Mexico Federico Gómez, following international guidelines for biomedical research involving humans (approval no. CIOMS-WHO 1993).

### 2.2. Samples Collection

Peripheral blood samples and bone marrow aspirates were collected after obtaining informed consent from the parents or guardians of patients, according to institutional protocols.

### 2.3. Mononuclear Cells Isolation

The mononuclear cells were isolated from peripheral blood and bone marrow aspirates by density gradient centrifugation with Lymphoprep™ (Axis-Shield), according to the manufacturer's protocol.

### 2.4. Immunophenotyping of NK Cell Subpopulations

Mononuclear cells (5 × 10^5^) from peripheral blood or bone marrow aspirates were plated in 96-well convex bottom plates and treated with blocking solution (0.1% NaN_3_, 2.0% FBS, 2% rabbit serum, and 5 mM EDTA) in the cold for 1 h. Cells were subsequently stained with monoclonal antibodies (mAb) at 4°C for 30 min; anti-CD56-PE (BD Biosciences) and anti-CD16-PerCP Cy5.5 (BioLegend, Inc.) were used to identify the different subpopulations of NK cells. To determine other populations of cells, anti-CD14-FITC (Santa Cruz Biotechnology, Inc.) was used to detect monocytes, anti-CD3-Pacific Blue for T-lymphocytes, and anti-CD19-PECy7 for B-lymphocytes (BD Biosciences). Cells were washed with staining buffer (0.1% NaN_3_, 2.0% FBS, and 5 mM EDTA) and fixed with 1% formalin. In total, 20,000 events from the lymphocyte regions were acquired using a FACS Aria II cytometer (BD Biosciences) after analysis with their respective autofluorescence and isotype controls and analyzed using FlowJo version XV (Tree Star, Inc.).

### 2.5. Enrichment of NK Cells

To determine the expression of TLRs in NK cells, three samples were randomly taken from each study group and CD56+ cells were enriched from peripheral blood and/or bone marrow mononuclear cells using an immunomagnetic separation kit (Miltenyi Biotec, GmbH), according to the manufacturer's protocol.

### 2.6. Determination of the Expression of TLRs in NK Cells

From the enriched CD56+ cells, slides were prepared using 1 × 10^4^ cells fixed with 4% regulated formalin for 15 min at room temperature (RT) and washed with 2% PBS-Tween 20 twice for 5 min. Cells were treated with Power Block™ Universal Blocker (BioGenex Laboratories) in a humidified chamber for 10 min at RT. The fixed cells were incubated with 10 specific anti-TLRs antibodies (Santa Cruz Biotechnology, Inc.) overnight at 4°C. After two washes with 2% PBS-Tween 20, cells were incubated with the secondary anti-goat FITC Ab for TLRs 1 to 9 and anti-mouse Ab FITC (Santa Cruz Biotechnology, Inc.) for TLR10 for 4 h at RT. Subsequently, anti-CD16-PE (Santa Cruz Biotechnology, Inc.) was added and incubated at 4°C overnight. Cells were then washed with 2% PBS-Tween, 3 times for 5 min, and the core marker DRAQ7 (Cell Signaling Technology, Inc.) was added for 20 min. For mounting, the slides were covered with mounting medium (PBS/Glycerol 1 : 1). In all cases, in the same slide, a spot was included for the corresponding isotype controls.

The article "NK Cell Subpopulation Is Altered and the Expression of TLR1 and TLR9 Is Decreased in Patients with Acute Lymphoblastic Leukemia" was published in 2021. Journal: J Oncol.

Cells were visualized using an Axiovert 100M LSM5 confocal microscope (Carl Zeiss AG) with a 40x/1.3x objective using immersion oil. A total of 10 photomicrographs were taken at 40x using a 1.8x zoom with the following configuration: 488 nm, 543 nm, and 633 nm lasers as well as LP 650, BP 505–530, and BP 560–615 filters. Images were taken consecutively using the same settings. The obtained images were analyzed using Zen 2009 (Carl Zeiss AG) and Image J (National Institutes of Health) [22].

### 2.7. Statistical Analysis

For statistical analysis, GraphPad Prism version 6 (GraphPad Software Inc.) was used. The medians of the frequencies of the different subpopulations of peripheral blood NK cells in patients with ALL were compared with a control group using a Mann–Whitney U test. As there were no control patients for bone marrow, a comparison was only performed against the peripheral blood NK cells of the ALL group.

To determine the differences, a semiquantitative analysis was performed by determining the fluorescence expression of the TLR in the 2D micrographs taken by confocal microscopy. The results were expressed as the medians of the MFI. The mean frequencies (MF) of peripheral blood NK cells (CD56+) from controls and ALL patients and bone marrow from ALL patients were calculated. The results of the expression of TLR 1 to 10 were expressed as the medians of the percentage of TLR+ CD16+ cells per 100 cells. Comparisons between each group were made using a Mann–Whitney U test. *P* < 0.05 was considered to indicate a statistically significant difference.

## 3. Results

### 3.1. Characteristics of the Patients

NK cells were analyzed in the peripheral blood and bone marrow aspirate from patients recently diagnosed with ALL, without treatment and/or infection. There were 13 males and 6 females with a mean age of 10.5 ± 4.6 years. In addition, control patients, six men, and four women with a mean age of 9.7 ± 3 years were included, of whom NK cells were analyzed in peripheral blood. The characteristics of each study group are summarized in Table 1.

The article "NK Cell Subpopulation Is Altered and the Expression of TLR1 and TLR9 Is Decreased in Patients with Acute Lymphoblastic Leukemia" was published in 2021. Journal: J Oncol.

### 3.2. Detection of NK^total^, NK^dim^, NK^bright^ Cells, and NK Supopulations in Patients with ALL

Analysis strategy to identify the different subpopulations of NK cells in patients with ALL.

The different subpopulations of NK cells from all samples were characterized as NK^total^ cells (CD14−, CD19−, CD3−, and CD56+) into NK^dim^ (CD56^low^, CD3−) and NK^bright^ (CD56^high^, CD3−) (Figure 1(a)). According to the CD56/CD16 expression, NK cells from all samples were subdivided into five subpopulations (I–V), as shown in Figure 1(a).

Representative flow cytometry results based on CD56/CD3 expression for each study group are shown in Figure 1(b).

The frequency of NK^total^ cells and their respective subpopulations (bright and dim) is expressed as the median ± percentage ranges with respect to the total lymphocyte population in Figure 1(c). The frequency of NK^total^ cells in peripheral blood of patients with ALL at diagnosis was significantly lower compared with the healthy controls (1.91% versus 4.89%; *P*=0.0075). Similarly, when comparing the results of NK^total^ cells of peripheral blood and bone marrow aspirates of patients with ALL, the percentage was significantly lower in the bone marrow (1.91% versus 0.635%; *P*=0.008; Figure 1(c)).

Conversely, the percentage of the NK^bright^ subpopulations in the peripheral blood was lower in the ALL group compared with the control group (0.08% versus 0.42%; *P*=0.0016), and there were no significant differences between the peripheral blood and bone marrow of the patients with ALL (0.08% versus 0.0455%; Figure 1(c)).

Likewise, the percentage of the NK^dim^ subpopulation in peripheral blood was lower in the ALL patients compared with the control group (2.2% versus 4.5%; *P*=0.0101); a significant decrease was also observed in the percentage of this subpopulation in bone marrow compared with the peripheral blood of patients with ALL (2.2% versus 0.53%, *P*=0.0052; Figure 1(c)).

### 3.3. Subpopulation of CD56− CD16+ NK Cells in Patients with ALL

After identification of NK cells based on the expression of CD56/CD3, they were stratified into five subpopulations, based on the differential expression of CD56 and CD16. NK^bright^ cells were subdivided into NK [CD56^high^ CD16−] (I) and NK [CD56^high^ CD16+] (II) cells, whereas NK^dim^ cells were subdivided into NK [CD56^low^ CD16−] (III) and NK [CD56^low^ CD16+] (IV) cells. A subpopulation of CD56− CD16+ (V) cells was also identified, as shown in Figure 2(a); peripheral blood results for a single control and a single patient with ALL and bone marrow results for a single patient with ALL are displayed.

The article "NK Cell Subpopulation Is Altered and the Expression of TLR1 and TLR9 Is Decreased in Patients with Acute Lymphoblastic Leukemia" was published in 2021. Journal: J Oncol.

The percentage of each subpopulation (I–V) found in the different groups is expressed as the median ± ranges with respect to the total NK^total^ cell [CD14−, CD19−, CD3−, CD56+, and CD16±] (Figure 2(b)); the medians of each of the groups of 10 controls and 10 or 9 patients with ALL are shown. In the peripheral blood of patients with ALL, there was a significant decrease in the percentage of subpopulation I (1.44% versus 3.43%; *P*=0.01) and IV (54.78% versus 74.40%; *P*=0.028) and an increase in subpopulation V (31.96% versus 13.99%; *P*=0.022) compared with the control group. It should be noted that there is an increase in subpopulation V [CD56− CD16+]. No significant differences were found between the percentages of each subpopulation between the peripheral blood and bone marrow aspirates of patients with ALL (Figure 2(b)).

### 3.4. TLRs Expression in NK CD16+ Cells in Patients with ALL

NK cells identified with CD16+ (red) belong primarily to the cytotoxic subtype of NK cells [NK^dim^ CD16+]; expression of all TLRs here can be seen in green, the nucleus in blue, and the colocalization of TLR with CD16 in yellow (Figure 3). The expression of TLR10 is reported in human NK [CD16+] cells for the first time.

The peripheral blood and bone marrow NK [CD16+] cells of pediatric patients with ALL, as well as those of healthy controls, differentially expressed the 10 TLRs, as shown in Figures 3–5, which show the representative results of one patient from each of the studied groups. In Figure 3, the results correspond to the colocalization of CD16 with TLR10. The expression of TLR10 is reported in human NK [CD16+] cells for the first time. In Figures 4 and 5, the results correspond to the colocalization of CD16 with the studied TLRs, 1 to 5 and 6 to 9, respectively.

The expression of each TLR was quantified as the MFI and the medians, and ranges of each group were plotted (Figure 6), which showed that the peripheral blood NK [CD16+] cells of patients with ALL exhibited lower TLR1 (297.8 versus 748.3; *P*=0.0042) and TLR9 expression (100.2 versus 190.7; *P*=0.0098) compared with the control group. Additionally, expression of TLR1 in bone marrow NK cells was increased compared with the peripheral blood cells of ALL patients (2,216 versus 297.8; *P*=0.0353). No significant differences in the expression of TLRs 2–8 and 10 were found between the groups. The TLRs with the highest level of expression in healthy controls were TLR1 and TLR2, whereas TLR9 exhibited the lowest levels of expression. Interestingly, the expression of TLR10 in the peripheral blood NK [CD16+] cells of patients and controls as well as in the bone marrow of patients with ALL was shown for the first time (Figure 6).

The article "NK Cell Subpopulation Is Altered and the Expression of TLR1 and TLR9 Is Decreased in Patients with Acute Lymphoblastic Leukemia" was published in 2021. Journal: J Oncol.

## 4. Discussion

A part of the present study was devoted to defining changes in the frequency of different NK cell subpopulations in total peripheral blood and bone marrow according to two different stratification strategies. The first was based primarily on the expression of CD56, called the “classic” phenotype, since it is accepted that there are at least two large populations of NK cells that correspond to the NK^bright^ (CD56^high^) and NK^dim^ (CD56^low^) phenotype [5, 23, 24]. The second strategy focused on subdividing NK cells into five subpopulations according to the differential expression of CD56 and CD16, the latter being a receptor that allows the different subpopulations to be discerned based on the degree of cytotoxic activity [6, 25], which is why they are termed “functional” phenotypes.

We observed that there was a significant decrease in the frequency of total NK cells [CD56+/CD3−] in peripheral blood lymphocytes of patients with ALL at the time of diagnosis compared with the control group. This result is consistent with previous studies in pediatric ALL patients [12, 26]. This behavior has also been observed in hematological disorders, such as myelodysplastic syndrome [27, 28] and acute myeloid leukemia [29], diseases characterized primarily by alterations present at the bone marrow level, both in the production of cells and in the microenvironment.

It was found that the total number of NK cells in the peripheral blood of ALL patients was lower than in the control group and the total number of NK cells in the bone marrow of the ALL patients was also lower, compared to the peripheral blood of the patients with ALL. These results agree with those obtained by Stabile et al. [26].

When comparing the total NK cell populations based on the classic phenotypic classification method, the subpopulation of NK^bright^ cells in the peripheral blood of patients with ALL was decreased compared with the control group and there was no difference with the bone marrow group. We also observed a decrease in NK^dim^ cells in the peripheral blood of patients with ALL compared with the control group and in the bone marrow was lower than in peripheral blood of patients with ALL. The proportion of the subpopulations in the peripheral blood and bone marrow of the ALL group was determined, and the 9 : 1 ratio (NK^dim^ : NK^bright^) was also observed in both cases and the control group. It was considered important to establish the changes in the proportion of the different subpopulations of NK cells since it is not enough to know whether or not there was a decrease in the amount of total NK cells [30].

The article "NK Cell Subpopulation Is Altered and the Expression of TLR1 and TLR9 Is Decreased in Patients with Acute Lymphoblastic Leukemia" was published in 2021. Journal: J Oncol.

The determination of the proportion of NK subtypes shows that the profile was predominantly cytotoxic.

The total NK cells were subdivided according to the CD56/CD16 expression to determine their functional phenotype, with the cells stratified into five subpopulations, which has been previously used for such a strategy [6, 25, 26].

Thus, NK^bright^ cells can be subdivided into two subpopulations: (I) NK^bright^ [CD56^high^ CD16^neg^] with a regulatory phenotype and (II) NK^bright^ [CD56^high^ CD16^low^] with a transitional phenotype. A lower percentage of subpopulation (I) was detected in the peripheral blood of the patients with ALL compared with the control group. There were no changes in the proportion of subpopulation (II) cells. When comparing the bone marrow aspirates with the peripheral blood, no significant differences were found in patients with ALL. Stabile et al. [26] did not divide NK^bright^ cells, classifying them as NK cells [CD56^high^ CD16±]. Contrary to the results of the present study, Stabile et al. [26] observed an increase in the total number but did not detect a notable change in the proportion of cells in the peripheral blood and bone marrow of ALL patients.

Similarly, NK^dim^ cells were divided into two subpopulations: (III) NK^dim^ [CD56^low^ CD16^neg^] and (IV) NK^dim^ [CD56^low^ CD16^high^] with a cytotoxic phenotype.

Regarding subpopulation III, there were no changes detected in its percentage or in the proportion with respect to total NK^dim^ counts, both in the peripheral blood and in the bone marrow. It was difficult to compare subpopulation III with the study by Stabile et al. [26], as their selection strategy highlights an NK subpopulation [CD56^low^ CD16^low^]; it is the set of subpopulation III [CD56^low^ CD16^neg^] proposed in the analysis and another extra subpopulation corresponding to the NK [CD56^low^ CD16^low^] that has received great attention in recent years. It has been shown that it is defined phenotypically and functionally as containing a high percentage of immature cells [NKG2A+ and CD57−], compared to their counterpart IV [CD56low CD16high], and exhibiting higher cytotoxic activity than subpopulation II [CD56bright CD16dim], but less than subpopulation III [CD56dim CD16neg] [31, 32]. It should be noted that, for the purpose of the present study, the extra subpopulation was not taken into account and only five subpopulations were reported.

There was a significant decrease in the proportion of subpopulation IV in the peripheral blood of patients with ALL compared with the control group. This proportion was similar in bone marrow, suggesting that their count was also decreased, as Stabile et al. [26] noted that the proportion of NK cells [CD56^low^ CD16^high^] was lower in both the bone marrow and peripheral blood of patients with ALL compared with the control group.

The article "NK Cell Subpopulation Is Altered and the Expression of TLR1 and TLR9 Is Decreased in Patients with Acute Lymphoblastic Leukemia" was published in 2021. Journal: J Oncol.

As for NK subpopulation (V) [CD56^neg^ CD16^high^], there was a greater amount of this subpopulation in the peripheral blood of patients with ALL compared with the healthy controls, and although there seemed to be an increase in the bone marrow, it was not possible to determine if this was significantly increased compared with healthy bone marrow. It should be noted that this is the first study where the increase of subpopulation (V) in disorders such as childhood ALL has been reported; to the best of our knowledge, as typically, the increase in this subpopulation has been associated with chronic viral diseases. In chronic viral diseases, it has been shown that subpopulation (V) cells exhibit low antiviral lytic activity, although they retain their ability to produce proinflammatory chemokines, which is why they have been termed dysfunctional [33]. In chronically ill patients with HIV, the virus causes an expansion of the proportion of these cells accompanied by a reduction in Siglec-7/NKG2A/CD57 and an increase in the NKG2C/KIR expression, which denotes a terminal phenotype [33]. To date, there are no studies showing how this subpopulation originates, what its role is in healthy or sick patients, and why their numbers expand in diseases such as leukemia.

In ALL, there are alterations in the receptors expressed by cytotoxic NK cells, which confer an inhibitory phenotype associated with impaired function, most notably IFN-y and TNF-α production and cytotoxicity. [12].

So that, the second portion of the present study was aimed at establishing the profile and level of expression of the 10 TLRs in NK cells with a cytotoxic phenotype [CD16^high^] in patients with ALL.

This part of the study was focusing on cytotoxic NK cells for two reasons: (i) NK cells were purified by positive selection through the CD56 marker, ruling out cells with the CD56^neg^ phenotype; and (ii) the frequency of NK^bright^ cells [CD56^high^ CD16^dim^] was considerably lower than NK cells with a cytotoxic phenotype [CD56^dim^ CD16^high^].

Until now, the expression of TLRs in NK cells has been partially reported by assessing changes at the mRNA level [19, 34]. The complete profile of TLRs at the protein level has not been determined to the best of our knowledge. Thus, the present study is the first to report, using confocal microscopy, the repertoire, and MFI of the 10 TLRs in NK cells from healthy individuals and ALL patients.

The article "NK Cell Subpopulation Is Altered and the Expression of TLR1 and TLR9 Is Decreased in Patients with Acute Lymphoblastic Leukemia" was published in 2021. Journal: J Oncol.

In healthy individuals, the MFI of TLRs 1 and 2 was higher compared with the other TLRs 3, 4, 5, 6, 7, 8, and 10; however, the expression levels of TLR9 were lower. It should be noted that the other TLRs did not show notable variations in their MFIs and were considered to have a mean level of baseline expression. These results bear some similarity with those reported at the mRNA level, since NK cells from healthy individuals have been shown to express elevated levels of TLR1 and very low levels of TLR9 [34, 35], followed by TLR2, TLR3, TLR5, and TLR6 [17, 18]. There are reports indicating that TLR4 and TLR7 (36) TLR8 and TLR10 [17, 34] exhibit low expression levels.

The peripheral blood and bone marrow NK cells in ALL patients expressed TLRs 1–10 with highly variable expression levels, but the expression of TLR1 and TLR9 was considerably lower in the peripheral blood of the group of patients with ALL compared to the control group, which may affect their recognition and activation capacity. Additionally, in the bone marrow of patients with ALL, the expression of TLR1 was considerably higher than that observed in the peripheral blood of patients with ALL and controls, a potentially interesting observation. To date, there are no studies examining the expression of these receptors in leukemic NK cells. However, there is a study where the expression of these receptors was analyzed in peripheral blood mononuclear cells (PBMC) from patients with ALL, observing a marked decrease in the expression of TLR1 and TLR9, but also of TLRs 3, 4, and 7 [36].

In other hematological cancers, such as acute myeloid leukemia (AML), the mRNA expression levels of TLR2 and TLR4, but not of TLR9, were increased, contrary to what was observed in ALL [37], and expression of TLR7 and 9 was decreased in chronic myeloid leukemia (CML) [38]. In chronic lymphocytic leukemia (CLL), there was an increase in the expression of TLRs 1, 2, 6, 7, 9, and 10 [38, 39]. This suggests that, in conditions such as chronic or acute leukemia, myeloid leukemia, or lymphoid leukemia, the profile and expression levels of TLRs may be abnormal. The individual study of the TLRs should be assessed in each cell lineage that participates in the antitumor response, in accessory cells of the medullary microenvironment, and in the leukemic cells, to detect the changes that could potentially promote or combat the antileukemic response. Different cell lines involved in the immune response are known to serve an important role in the early defense against MAMPs and/or against PAMPs via TLRs, promoting the inflammatory response.

The article "NK Cell Subpopulation Is Altered and the Expression of TLR1 and TLR9 Is Decreased in Patients with Acute Lymphoblastic Leukemia" was published in 2021. Journal: J Oncol.

In this study, the NK cells from peripheral blood of patients with leukemia show a significant decrease in the expression of TLR1, but not of TLR2. This suggests that the response to the TLR1/2 ligands may not be effective.

Regarding TLR9, CpG-DNA is reported to bind to the KIR3DL2 receptor (activator receptor) for transportation to an endosomal compartment, where it is presented to TLR9 for its activation as a unique mechanism of NK cells, which conditions its potential response to TLR9 ligands [40]. In our study, NK cells from peripheral blood of patients with ALL exhibited a decrease in the expression of TLR9; perhaps this decrease may also be related to the inhibitory phenotype of the NK cells.

It is possible that the leukemic microenvironment and even the leukemic cells themselves cause decreased expression of TLR activators in NK cells through a mechanism similar to that described by Rouce et al. [12] where it has been shown that leukemia cells induce the TGF-*β*/SMAD pathway in NK cells of leukemic patients, causing their dysfunction and low cytotoxic activity.

There is no information on whether the alteration in the expression and/or function of TLRs is due to the leukemic microenvironment (leukemic niche), to the leukemic cells, or if there are alterations at the genetic level that may condition the response in NK cells or other cells of the immune system to TLR ligands.

NK cells from bone marrow, compared with those from peripheral blood in patients with ALL, showed a greater than double increase in the level of expression of TLR1. Since there is no information regarding the differences between the expression profiles of TLRs in peripheral blood cells compared to those in bone marrow, it is not possible to explain this finding.

In the present study, the profile and expression levels of 10 TLRs were detected, data that will serve as a reference to determine the ligands of TLRs that could be useful to increase cytotoxic activity and the activating phenotype that characterizes NK cells. It has been shown that the ligands of TLRs can be used as a promising therapeutic alternative for several types of cancer, some of which are already in clinical trials [41].

## 5. Conclusion

Pediatric patients with ALL exhibited a significant decrease in the total frequency of NK cells in the peripheral blood and in the bone marrow, in addition to presenting alterations in the distribution of the subpopulations of NK cells. This alteration in subpopulations may condition the immune response mediated by these cells as the proportion of the main functional phenotypes, regulatory and cytotoxic, was decreased, whereas the dysfunctional phenotype was considerably increased as a consequence of the leukemic process.

The article "NK Cell Subpopulation Is Altered and the Expression of TLR1 and TLR9 Is Decreased in Patients with Acute Lymphoblastic Leukemia" was published in 2021. Journal: J Oncol.

NK cells of ALL patients expressed all 10 TLRs recognized in humans at the protein level; the expression levels of TLR1 and TLR9 were decreased in peripheral blood patients with ALL.

The expression of TLR1 was higher in the bone marrow NK cells compared with the peripheral blood NK cells in patients with ALL, which may represent the importance of the sentinel role of this receptor at the bone marrow level.

## Figures and Tables

**Figure 1:** Characterization of NK cell subpopulations using flow cytometry. (a) First, the NK^total^ cells [CD14−, CD19−, CD3−, and CD56+], NK^dim^ [CD56^low^ CD3−], and NK^bright^ [CD56^high^ CD3−] were detected, and subsequently, the subpopulations (I–V) based on the expression of CD56/CD16 were detected. (b) Identification of all NK cells in the peripheral blood of controls and ALL patients, and in the bone marrow of ALL patients. Representative flow cytometry results based on CD56/CD3 expression for each study group are shown. (c) Graphs showing the percentage of NK^total^, CD56^bright^, and CD56^dim^ cells (median ± ranges) in the peripheral blood of 10 controls and 9 patients with ALL and in the bone marrow of 10 patients with ALL. ^*∗*^*P* < 0.05. NK, natural killer; ALL, acute lymphoblastic leukemia.

**Figure 2:** Determination of NK cell subpopulations using the CD56/CD16 phenotype. (a) Histograms of subpopulations of NK cells in the controls and ALL patients in the peripheral blood and in the bone marrow of ALL patients; peripheral blood results for a single control and a single patient and bone marrow results for a single patient are displayed. NK^bright^ cells can be subdivided into (I) NK [CD56^high^ CD16−] and (II) NK [CD56^high^ CD16+]; NK^dim^ cells can be subdivided into (III) NK [CD56l^ow^ CD16−], (IV) NK [CD56^low^ CD16+], and (V) NK [CD56− CD16+] cells. (b) Graph showing the percentage (median ± ranges) in each subpopulation (IV) with respect to the total NK^total^ count [CD14−, CD19−, CD3−, CD56+, and CD16±] in the peripheral blood of 10 controls and 9 patients with ALL and in the bone marrow of 10 patients with ALL; the medians of each of the groups are shown. ^*∗*^*P* < 0.05. NK, natural killer; ALL, acute lymphoblastic leukemia.

**Figure 3:** Expression of TLR10 in cytotoxic NK cells of controls and patients with ALL. Representative micrographs of TLR10-positive NK cells (red) determined in the peripheral blood of controls and ALL patients and in the bone marrow of ALL patients. Nuclei were differentiated using DRAQ7 (blue). A merge of the micrographs with the bright field image is also shown. Magnification, x40. TLR, Toll-like receptor; NK, natural killer; ALL, acute lymphoblastic leukemia.

The article "NK Cell Subpopulation Is Altered and the Expression of TLR1 and TLR9 Is Decreased in Patients with Acute Lymphoblastic Leukemia" was published in 2021. Journal: J Oncol.

**Figure 4:** Expression of TLRs 1–5 in cytotoxic NK cells from controls and ALL patients. Representative micrographs of NK cells (red) positive for TLRs 1, 2, 3, 4, and 5 (green) determined in the peripheral blood of controls and patients with ALL and in the bone marrow of patients with ALL. Nuclei were differentiated using DRAQ7 (blue). TLR, toll-like receptor; NK, natural killer; ALL, acute lymphoblastic leukemia.

**Figure 5:** Expression of TLRs 6–9 in cytotoxic NK cells from controls and ALL patients. Representative micrographs of NK cells (red) positive for TLRs 6, 7, 8, and 9 (green) determined in the peripheral blood of controls and patients with ALL and in the bone marrow of patients with ALL. Nuclei were differentiated using DRAQ7 (blue). TLR, toll-like receptor; NK, natural killer; ALL, acute lymphoblastic leukemia.

**Figure 6:** Graph of the MFI of the 10 TLRs evaluated in NK cells obtained from peripheral blood of 10 controls and 9 patients with ALL and from the bone marrow of 10 patients with ALL. Micrographs obtained using confocal microscopy. Magnification, x40. Images were analyzed using Zen 2009. ^*∗*^*P* < 0.05. MFI, mean fluorescence intensity; TLR, Toll-like receptor; NK, natural killer; ALL, acute lymphoblastic leukemia.

**Table 1:** Demographic characteristics of patients and controls.

	Healthy donors	ALL patients
Characteristic	Peripheral blood	Peripheral blood
	Control	ALL
No. of cases	10	9
Age range (years)	9.7 ± 3	10.5 ± 4.6
Sex (M : F)	6 : 4	7 : 2
ALL immunophenotype	N/A	Pro-B = 3 Pre-B = 3 *T* = 1 Not classifiable = 2
Blast infiltration (%)	N/A	78 ± 0.12%
Risk classification	N/A	High= standard = 1

## Data Availability

The datasets used and/or analyzed during the current study are available from the corresponding author on reasonable request.
